# Variations and Determinants of Anemia among Reproductive Age Women in Five Sub-Saharan Africa Countries

**DOI:** 10.1155/2021/9957160

**Published:** 2021-08-05

**Authors:** Josephine Nti, Seth Afagbedzi, Frances Baaba da-Costa Vroom, Noor Akma Ibrahim, Chris Guure

**Affiliations:** ^1^Department of Biostatistics, School of Public Health, University of Ghana, Accra, Ghana; ^2^Institute for Mathematical Research, Universiti Putra Malaysia, Serdang, Selangor, Malaysia

## Abstract

**Background:**

The Ghana Demographic and Health Survey 2014 report indicates that anemia among women in their reproductive age in the country stood at 42 percent, making it a severe public health problem according to the World Health Organization (WHO) classification. WHO Global Observatory data indicates that some sub-Saharan African countries have been able to reduce the prevalence of anemia among women of reproductive age compared to Ghana in 2016. To inform policy decisions, data from the Demographic and Health Surveys 2014–2018 were analyzed to determine the disparities in the prevalence of anemia and related factors among women of reproductive age in Ghana, Ethiopia, Uganda, Tanzania, and Rwanda.

**Methods:**

This research utilized data from the Demographic and Health Surveys 2014, 2016, 2014-2015, 2015-2016, and 2016 from Ghana, Ethiopia, Rwanda, Tanzania, and Uganda, respectively. Respondents were women aged between 15 and 49 years. Hemoglobin levels were measured by HemoCue hemoglobin meter. 45,299 women data were extracted from the five countries with 4,644, 14,923, 6,680, 13,064, and 5,988 from Ghana, Ethiopia, Rwanda, Tanzania, and Uganda, respectively. Association between anemia and selected predictive variables was assessed using Pearson's chi-square test statistic. Poisson regression with robust standard errors was used to estimate the prevalence rate ratios of developing anemia. The deviance goodness of fit test was employed to test the fit of the Poisson model to the data set.

**Results:**

There was a statistically significant difference in prevalence of 1,962 (42.3%), 3,527 (23.6%), 1,284 (19.3%), 5,857 (44.8%), and 1,898 (31.7%) for Ghana, Ethiopia, Rwanda, Tanzania, and Uganda, respectively, *χ*^2^ = 2,181.86 and *p* value < 0.001. Parity, pregnancy status, and contraceptives significantly increased the prevalence rate ratio of a woman developing anemia. Women in Ethiopia with a parity of six or more were 58% more likely to develop anemia than those with parity of zero. Tanzanian women who were pregnant had a 14% increased rate ratio of developing anemia. Factors that significantly decreased anemia in this study were wealth index, women's age, and women's highest level of education. Women who were in the higher education category in Ethiopia were 57% less likely to develop anemia. Ugandan women in the richest category of the wealth index were 28% less likely to develop anemia. Rwandan women in the middle category of the wealth index were 20% less likely to develop anemia. Women who were within the 45-49 age category in Ethiopia were 48% less likely to develop anemia.

**Conclusion:**

The individual country governments should encourage the implementation of increasing female enrollment in higher education. Women in their reproductive age should be encouraged to use modern contraceptives to reduce their anemia prevalence.

## 1. Background

Anemia was identified as one of the major public health problems in developing countries. It is reported to account for three-quarters of a million deaths per year in Africa and Southeast Asia (World Health Organization, 2015). World Health Organization (WHO) data shows that approximately 10.8 million women in Africa and 9.7million women in the Western Pacific are anemic [1]. The prevalence may be as high as 42-61% in developing countries in malaria-endemic areas such as Ghana [2]. Worldwide prevalence of anemia according to [3]) has been estimated according to regions and population groups. In the analysis, women and young children were mostly vulnerable to anemia. The proportion of women and children who develop anemia is high in the African region. About 48% of nonpregnant women and 68% of preschool children are anemic [3].

According to Qiuyue et al. [4], anemia is seen as an important public health problem throughout the world, particularly in developing countries with the overall prevalence of severe anemia (hemoglobin level less than 8.0 g/dl) among nonpregnant women of reproductive age being 1.1%. Prevention of anemia in nonpregnant women could improve their health status when the same women get pregnant, eventually contributing to the reduction of both maternal and perinatal mortalities [4]. The consequences of morbidity associated with chronic anemia extend to loss of productivity from impaired work capacity, cognitive impairment, and increased susceptibility to infection, which also exerts a substantial economic burden [5].

According to the World Health Organization 2016, Global Health Observatory Data on the prevalence of anemia among women in their reproductive age for the years 1990 to 2016, some sub-Saharan African countries had improved on reducing anemia prevalence compared to others. Information on anemia prevalence for five selected countries, namely, Ethiopia, Rwanda, Uganda, Tanzania, and Ghana, indicate that four out of these five countries have been able to reduce anemia prevalence among women in their reproductive ages. This percentage point reduction is between 10% and 28% over the last twenty-six years except for Ghana, which had a reduction in prevalence of less than 10%. The prevalence of anemia among women in the five countries in 1990 and 2016, respectively, was as follows: Ghana (55.3% and 46.4%), Ethiopia (47.3% and 23.0%), Rwanda (32.3% and 22.0%), Uganda (44.3% and 29.0%), and Tanzania (50.9% and 37.0%). This information shows that Ghana can learn lessons from other countries to reduce its prevalence of anemia among women in their reproductive age. This will be possible if Ghana acclimatizes the kind of interventions that these other four countries have used to reduce the prevalence of anemia among women. Analysis of datasets from surveys of these countries will help to identify factors that are reducing the prevalence of anemia among women in these countries than others since at a global level, anemia prevalence is a useful indicator to assess the impact of highly effective interventions and to track the progress made towards the goal of reducing anemia. To make a meaningful analysis and interpretation, it was necessary to analyze the datasets of Demographic and Health Surveys available for these five countries.

The WHO 2016 Observatory report about the prevalence of anemia in these African countries informed the decision to include these countries as part of this study. Ghana and Tanzania fell within the severe public health significance (≥40.0%) level. Ethiopia and Uganda fell under moderate public health significance (20-39.9%). Rwanda was the only country with mild public health significance (5-19.9%). This study finds it imperative to determine the variations in prevalence of anemia among women of reproductive age across these selected countries (Ghana, Ethiopia, Rwanda, Uganda, and Tanzania) and identify determinants that could influence its high prevalence among women in their reproductive age in order to reduce its adverse effects nationally.

## 2. Methods

### 2.1. Data Source

The secondary data were obtained from the Demographic and Household Surveys of five sub-Saharan African countries: Ghana, Ethiopia, Rwanda, Tanzania, and Uganda, between 2014 and 2016 through the DHS programme data access portal. All study participants were nationally represented and selected from all regions/provinces of each country and stratified according to urban and rural areas. A review of all the survey reports states that a two-stage sampling design was used for all the selected countries. The first stage of this had to do with the selection of enumeration areas (EA), the primary sampling unit, from an updated master sampling frame constructed from a previous population census. In the second stage, households were systematically selected from all the clusters to provide adequate estimates for key indicators with acceptable precision. The variables for this analysis were extracted from the Demographic and Health Surveys from the five countries. The total number of eligible women interviewed for Ghana, Ethiopia, Rwanda, Uganda, and Tanzania was 4,644, 14,923, 6,680, 5,988, and 13,064, respectively.

### 2.2. Dependent Variable

Anemia cut-off points used in this study were those recommended by WHO for nonpregnant and pregnant women [3, 6]. Any anemia was defined as hemoglobin (Hb) ≥ 12.0 g/dl in nonpregnant women and Hb ≥ 11.0 g/dl in pregnant women. Mild anemia was defined as Hb level between 11.0 and 11.9 g/dl among nonpregnant women and between 10.0 and 10.9 g/dl among pregnant women. Moderate-to-severe anemia was defined as Hb lower than 10.9 g/dl and 9.9 g/dl in both nonpregnant and pregnant women. The dependent variable used in this study, named anemia status, involved grouping of the categories of the variable anemia level into two categories, that is, anemia (mild, moderate, and severe) and no anemia (Hb higher or equal to 11.0 g/dl in pregnant women and Hb higher or equal 12.0 g/dl in nonpregnant women).

### 2.3. Statistical Methods

In all the analysis, we adjusted for the complex nature of the survey design by accounting for clustering, stratification, and weighting. Due to the comparisons and combination (pooled data) of different surveys from different countries, with different target population sizes, the weights were denormalized. This was done by dividing the women standard weights and their total number in each country by the respective survey sampling fraction. The analysis was performed using descriptive, bivariate, and multivariate regression procedures. Descriptive statistics was done to explore the dependent and independent variables of interest. Bivariate analysis with Pearson's chi-square test was used to assess significant associations between the dependent (anemia status) and independent variables. These variables are age of respondent, type of place of resident, highest level of education, wealth index, partner's educational level, woman's occupation, partner's occupation, parity, health insurance use, contraceptive use, bed net use, marital status, age at first birth, and pregnant at the time of study. Poisson regression with robust standard error was used to approximate the prevalence rate ratio (PRR) of being anemic for variables that showed some level of significance at the bivariate level of analysis, a powerful statistical modelling method that allows the incorporation of explanatory variables at different levels of the hierarchy. According to Barros et al. [7], Poisson regression with a robust standard error has proven to be a better alternative to logistic regression, especially for cross-sectional studies with binary outcomes. This is because Poisson produces accurate estimates in the form of prevalence rate ratios that are more interpretable and easier to communicate to nonspecialists than the odds ratios of logistic regression [7]. An additional advantage of Poisson regression is that the estimates are relatively robust to omitted covariates in contrast to logistic regression [8]. The issue of overdispersion (large variability), which affects the standard errors and consequently the confidence intervals in Poisson regression, is rectified when they are estimated using the sandwich variance estimator [8–10]. Variables that showed statistical significance and were seen as potential confounders were adjusted for. Variables like type of place of residence, pregnant at the time of study, and marital status, which did not show a significant association at the bivariate level, were included because they were found in the literature to be significantly associated with the outcome (anemia) of interest. We assessed the effect of interactions between the independent variables, and none was significant nor improved the performance of the model fit. Multicollinearity was also examined, and there was no collinearity between variables. Statistical significance was set at a cut-off value of *p* < 0.05 with a confidence level of 95%. The deviance goodness of fit test was specified to test whether the Poisson model fits the individual country specific data well as well as the pooled data. All analyses were done in Stata 15 and graphs generated with Excel 2013. All estimates were analyzed using the Stata Survey Analysis tool where primary sampling units, stratification, and weights are accounted for.

## 3. Results

A total of 45,299 women (15-49 years) data were included in this study consisting of five countries, of which 4,644 (10.3%) women were from Ghana, 14,923 (32.9%) were from Ethiopia, 6,680 (14.8%) from Rwanda, 13,064 (28.8%) from Tanzania, and 5,988 (13.2%) from Uganda. Ethiopia was the country with the highest percentage of richest women of 30.0% and a lowest percentage of 21.8% for Ugandan women. Rwanda had the highest percentage of 19.6% for the poorest women, and Ethiopia had the lowest percentage of 16.9% for the poorest women of reproductive age. Rwanda showed a highest percentage of 80.2% for rural dwellers while Ghana had the lowest percentage of 46.1% for rural dwellers. The highest percentage of urban dwellers was 53.9% and found in Ghana, and the lowest percentage of 19.8% for urban dwellers was recorded in Rwanda.

Type of place of residence and bed net use were not statistically significant at the bivariate level of analysis when all five country data were combined. However, Ethiopia, Rwanda, and Uganda were the countries that showed statistical significance for the type of place of residence just like all the five countries' combined data. All individual countries showed a statistically significant association with bed net use.

### 3.1. Variations in Prevalence of Anemia among Women in the Five Selected Countries

The results of this analysis showed that the prevalence of anemia among the five countries was significantly different with *χ*^2^ = 2181.86 and a *p* value < 0.001 (Figure 1).

Country of residence was statistically significantly associated with anemia status at the bivariate level. Women who lived in Ethiopia, Rwanda, and Uganda showed a statistically significantly decreased crude prevalence rate ratio of CPRR: 0.56, CI (0.52, 0.59)^∗∗∗^; CPRR: 0.45, CI (0.43, 0.48)^∗∗∗^; and CPRR: 0.75, CI (0.71, 0.79)^∗∗∗^, respectively, while women from Tanzania were 6% more likely to become anemic compared to Ghana. Adjusted analysis showed that the rate ratio among Ethiopia and Ugandan women was to decrease by 38% and 23% compared to Ghana.

### 3.2. Variations in Prevalence of Anemia among Women According to Residence in the Five Selected Countries

Figure 2 shows the distribution of women (15-49 years) who were anemic according to the type of place of residence among the five countries and all countries put together. All individual countries showed an increased anemia prevalence of women living in rural areas than women in urban areas except for all the countries put together that showed an increased prevalence in women in urban areas than women in rural areas. Apart from Tanzania, Ghana had the highest anemia prevalence for both women in urban and rural areas that were 41.8% and 43.1%, respectively. Rwanda had the lowest prevalence of anemia for both women in urban and rural areas being 16.3% and 19.9%, respectively.

### 3.3. Factors that Significantly Increased the Prevalence of Anemia among the Selected Countries

The highest prevalence of anemia according to age groups varied across the selected countries. Ghana, Ethiopia, Tanzania, and all countries put together had a statistically significant association between a woman's age and anemia status.  Table 1 shows that the 15-19 year's category recorded the highest anemia prevalence of 47.7% and 47.3% for both Ghana and Tanzania, respectively. Women who were 30-34 years had the highest prevalence of 26.6% in Ethiopia. When all five countries were put together, the highest prevalence was found among women who were 40-44 years of age. However, using the age category 15-19 years as the reference category at the multivariate level, only Ethiopia showed a significant increased prevalence rate ratio of PRR: 1.33 at 95% CI (1.15, 1.54)^∗∗∗^ for age category 30-34 years at the unadjusted level in Table 2.

Women who lived in the rural areas of Ethiopia, Rwanda, and Uganda had a statistically significantly increased anemia prevalence of 25.4%, 19.9%, and 33.2%, respectively. Women in the rural areas of Ethiopia had a statistically significant 1.49 factor of getting anemia compared to their urban counterparts while rural women in Uganda had 21% increased rate ratio of getting anemia compared to their urban folks. Adjusted analysis showed a 15% increased rate ratio of rural women in Ethiopia.

Anemia status and wealth index showed a statistically significant association for all five countries as well as the combined dataset. All five countries recorded the highest anemia prevalence among the poorest category, except for Ghana which showed the highest prevalence of 50.5% among the poorer women category. The highest anemia prevalence recorded among the other four countries was 32.3% for Ethiopia, 24.8% for Rwanda, 48.5% for Tanzania, and 40.6% for Uganda. When all five countries were put together, the highest anemia prevalence was still among the poorest category with a prevalence of 38.5%. The multivariate level of analysis observed a statistically significant increase in the prevalence rate ratio of 21% among the poorer women category for Ghana.

Ghana, Ethiopia, and Rwanda recorded their highest prevalence among the category of women who did not have any intention of using modern contraceptives. The prevalence was 44.1% for Ghana, 27.9% for Ethiopia, and 22.0% for Rwanda. However, results from Tanzania and Uganda showed the highest prevalence for both countries among women who intended to use modern contraceptives later with a prevalence of 49.3% for Tanzania and 36.8% for Uganda.

Ghana and Tanzania recorded a statistically significantly increased prevalence of 44.8% and 47.2%, respectively, for women who used bed nets. Tanzanian women who used bed nets had a 1.21 factor of developing anemia. Women in Ethiopia with a parity of six or more had a 1.58 factor of developing anemia than those with a parity of zero. Tanzanian women who were pregnant had a 14% increased rate ratio of developing anemia compared to those who were not pregnant.

### 3.4. Factors that Significantly Decreased the Prevalence of Anemia among the Selected Countries

Age of the woman had a statistically significant association with anemia status in Ghana, Ethiopia, and Tanzania. Women in Ghana who fell within the 45-49-year category recorded the lowest prevalence of 37.5%. Among women in Ethiopia, those who were 15-19 years of age recorded the lowest prevalence of 19.9%. The lowest anemia prevalence in Tanzania was 40.8% among 30-34 years. Women in Ethiopia found among the category of 45-49 years had a 48% lower rate ratio of developing anemia than those who were 15-19 years, whereas Tanzanian women in the same (45-49) year category had a 18% lower rate ratio to get anemia.

Wealth index showed a statistically significant association with anemia status for all the individual countries as well as all five countries put together. The richer women category recorded the lowest prevalence of 37.2%, 16.1%, and 41.2% for Ghana, Rwanda, and Tanzania, respectively. Comparing between Ethiopia, Rwanda, and Uganda, the richest category of women in Ethiopia had a 37% lower rate ratio of developing anemia compared to their poorest women category. The richest category of Rwanda showed a 25% decreased rate ratio of getting anemia. Similarly, women among the richest category in Uganda had a 28% decreased rate ratio of developing anemia. Rwanda and Uganda showed a statistically significantly low prevalence for women who used bed nets with a *p* value < 0.05.

A woman in Ethiopia and Uganda had a 38% and 23% decreased rate ratio of developing anemia compared to their counterparts in Ghana, respectively. Women in Uganda were 23% less likely to develop anemia compared to women in Ghana. The deviance goodness of fit test showed that the Poisson model did fit all the data well. The *p* values for the individual country analysis and that of the pooled data were highly insignificant (*p* value = 1.00).

## 4. Discussion

### 4.1. Variations in the Prevalence of Anemia among Women in the Five Selected Countries

The objectives of this study were to examine the variations and factors that either increase or decrease anemia prevalence in selected African countries based on the burden of the disease and availability of DHS data. From the analysis, we observed a significant variation in the prevalence of anemia for all countries (*p* value < 0.001). Tanzania recorded the highest prevalence of anemia while Rwanda had the lowest prevalence. The overall prevalence on the combined data was 32.1%.

### 4.2. Factors that Significantly Increased the Risk of Anemia among the Selected Countries

The results show that factors like marital status and contraceptive use significantly increased the rate ratio of a woman getting anemia across all five countries. Different factors increased the rate ratio of a woman developing anemia in some countries. In Ghana, wealth index, partner's occupation, age at first birth, and contraceptive use were factors that increased a woman's likelihood of getting anemia. Women who were poorer were more likely to develop anemia in Ghana. This is in line with the study by Bentley and Griffiths [3] in India while it contradicts studies done by Ngnie-Teta et al. [11] and Ghose and Yaya [12] where it was observed that women in the middle wealth index category rather had the increased rate ratio of anemia [11, 12]. Women whose partners' occupation was sales and those who worked in the agricultural sector had a higher rate of developing anemia. Women in Ghana whose age at first birth was between 25 and 29 years and those greater or equal to 30 years had increased factors to develop anemia. In Rwanda, marital status and contraceptive use statistically significantly increased the woman's rate ratio of developing anemia. Women who did not intend to use modern contraceptives at all and those who intend to use modern contraceptives later all had an increased rate ratio to develop anemia. This is in line with two studies on modern contraceptive use [13, 14].

When all the five countries were put together, partner's occupation, marital status, and contraceptive use increased the rate ratio of a woman developing anemia. Women who intended to use modern contraceptives later had a 1.51 factor of developing anemia than those who used modern contraceptives.

### 4.3. Factors that Significantly Decrease the Risk of Anemia among the Selected Countries

Factors that significantly decreased a woman's prevalence rate of getting anemia were women's age, education, and occupation. Women with secondary and higher educational levels were 5% and 21% less likely to have anemia. This could be attributable to the fact that being educated could increase or improve the woman's knowledge on danger signs, prevention, cure, and interventions for anemia to make the right choices and prevent anemia.

In Rwanda, bed net use and wealth index significantly decreased a woman's rate ratio of getting anemia. This is supported by a study conducted by [15] but in contrast to a study conducted in Timor-Leste on women in their reproductive age where there was no association between bed net use and anemia prevalence [16]. Women who used bed nets in Rwanda were 8% less likely to develop anemia. For all countries put together, women's occupation significantly decreased the prevalence rate ratio of getting anemia. Women who lived in Ethiopia, Rwanda, and Uganda showed a statistically decreased rate ratio compared to Ghana.

### 4.4. Lessons Ghana, Tanzania, Ethiopia, and Uganda Can Learn from

All these countries can aspire to reduce anemia prevalence from within the severe and moderate public health problem category to at least a mild public health category like Rwanda.

Comparing these countries to Rwanda, poorer women in Rwanda had a decreased prevalence rate ratio of anemia than their counterparts in the other countries. In addition, bed net use in Rwanda decreased significantly the rate ratio of anemia. Since bed net use was seen to significantly decrease the rate ratio of anemia in Rwanda, there is the need for the private sector to collaborate with individual country's governments through advocacy campaigns and intensify education on the appropriate use of this intervention in addition to its funding.

Women who did not intend to use any form of modern contraceptives had an increased prevalence rate ratio of anemia. There is therefore the need for advanced research to identify specific types of modern contraceptives that will significantly reduce the rate ratio of a woman developing anemia with minimal or no side effects. This is to educate women appropriately and encourage the use of modern contraceptives in reducing the prevalence of anemia.

## 5. Conclusions

The analysis found a high prevalence in Ghana and Tanzania, and all two fell within the severe public health significance category. Ethiopia and Uganda also fell within the moderate public health significance category with only Rwanda within the mild public health significance category. The study found wealth index, contraceptive use, partner's occupation, and age at first birth to be significantly increasing the risk of getting anemia. Woman's educational status and women's occupation in Ghana were found to decrease significantly the risk of anemia. Comparing Ghana to Rwanda, poorer women in Rwanda had a decreased risk of anemia than their counterparts in Ghana. Additionally, bed net use in Rwanda decreased significantly the risk of anemia. Since bed net use was seen to significantly decrease the risk of anemia, there is the need for the private sector to partner the Ghana government through advocacy campaigns to intensify the education on the appropriate use of this intervention in addition to its funding.

## Figures and Tables

**Figure 1:** Prevalence of anemia among women (15-49 years) in five sub-Saharan African countries and all five countries put together using DHS data from 2014 to 2018.

**Figure 2:** Distribution of women (15-49 years) who had anemia according to the type of place of residence among five sub-Saharan African countries using DHS data from 2014 to 2018.

**Table 1:** Prevalence of anemia in women aged 15–49 years using data from the Demographic and Health Surveys of five sub-Saharan African countries from 2014 to 2018.

	Ghana *N* = 4,644	Ethiopia *N* = 14,923	Rwanda *N* = 6,680	Tanzania *N* = 13,064	Uganda *N* = 5,988	All five *N* = 45,299
	Anemic	Anemic	Anemic	Anemic	Anemic	Anemic
Age of Res.						
15-19	383 (47.7)	631 (19.9)	260 (18.7)	1358 (47.3)	450 (32.9)	3082 (32.1)
20-24	374 (46.9)	627 (23.8)	240 (19.6)	1131 (46.3)	411 (33.7)	2784 (33.5)
25-29	308 (39.6)	693 (24.4)	208 (18.0)	901 (42.8)	273 (27.4)	2382 (30.3)
30-34	270 (38.5)	597 (26.6)	184 (17.9)	704 (40.8)	256 (31.0)	2011 (30.8)
35-39	254 (39.2)	442 (24.1)	155 (19.5)	739 (46.0)	203 (31.0)	1793 (32.4)
40-44	222 (44.3)	312 (25.4)	121 (19.8)	602 (45.0)	184 (33.5)	1442 (34.0)
45-49	156 (37.5)	225 (22.9)	116 (24.1)	422 (43.2)	121 (32.5)	1040 (32.2)
Type of place of residence						
Urban	1047 (41.8)	539 (17.0)	217 (16.3)	2083 (44.5)	423 (27.4)	4308 (32.6)
Rural	921 (43.1)	2988 (25.4)	1068 (19.9)	3774 (45.0)	1475 (33.2)	10224 (31.9)
Res. Educ.						
No Educ.	412 (45.5)	2002 (27.7)	179 (22.5)	979 (51.3)	212 (36.7)	3786 (33.2)
Primary	377 (44.7)	1136 (21.7)	824 (19.1)	3609 (44.5)	1090 (31.7)	7036 (32.0)
Secondary	1093 (41.6)	298 (17.8)	243 (17.6)	1204 (41.8)	466 (30.4)	3303 (32.7)
Higher	86 (32.1)	91 (11.5)	38 (20.7)	65 (41.4)	129 (29.7)	409 (22.3)
Wealth index						
Poorest	345 (43.6)	863 (32.3)	324 (24.8)	1079 (48.5)	437 (40.6)	3048 (38.5)
Poorer	403 (50.5)	689 (25.3)	265 (20.1)	1042 (46.2)	351 (32.9)	2749 (33.7)
Middle	439 (45.2)	686 (23.7)	236 (18.8)	1060 (45.9)	343 (30.6)	2763 (32.4)
Richer	382 (37.2)	625 (21.0)	202 (16.1)	1147 (41.2)	389 (31.8)	2746 (29.6)
Richest	398 (37.7)	664 (17.4)	259 (16.6)	1528 (43.7)	378 (25.2)	3228 (28.2)
Preg. at time of study						
No	1816 (42.2)	3212 (23.2)	1170 (18.9)	5218 (43.7)	1663 (30.9)	13077 (31.4)
Yes	152 (44.6)	317 (29.1)	115 (23.4)	639 (57.1)	235 (38.2)	1457 (40.0)
Health Ins.						
No	755 (43.2)	3392 (24.0)	-	5393 (45.4)	1878 (31.7)	11420 (33.9)
Yes	1212 (41.9)	135 (16.8)	-	463 (39.5)	20 (28.6)	1830 (37.1)
Marital status						
Never married	664 (44.5)	667 (17.7)	485 (19.1)	1463 (44.2)	467 (30.6)	3747 (29.7)
Married	797 (40.7)	2524 (26.3)	387 (16.8)	2628 (44.8)	581 (31.3)	6918 (32.1)
Living with partner	300 (42.9)	48 (23.8)	238 (21.1)	999 (44.7)	557 (31.0)	2143 (35.3)
Widowed	50 (42.5)	89 (21.5)	76 (27.5)	170 (45.9)	70 (41.9)	455 (34.0)
Divorced	65 (43.5)	139 (18.9)	37 (20.4)	295 (48.0)	17 (33.7)	552 (32.0)
Not with partner	92 (41.1)	61 (27.5)	61 (25.0)	301 (43.8)	204 (34.9)	719 (36.7)
Partner's Educ.						
No Educ.	305 (47.8)	1281 (28.4)	166 (21.4)	506 (51.1)	77 (34.0)	2334 (32.7)
Primary	101 (39.2)	941 (25.7)	532 (18.9)	2442 (44.0)	615 (32.6)	4631 (32.7)
Secondary	707 (39.3)	206 (22.5)	75 (18.5)	566 (44.2)	292 (28.9)	1844 (34.1)
Higher	158 (41.4)	117 (18.1)	22 (17.4)	109 (41.8)	120 (28.3)	526 (28.6)
Do not know	34 (42.0)	28 (36.4)	4 (26.1)	5 (42.6)	36 (31.6)	107 (35.7)
Woman's Occup.						*N* = 45281
Not working	517 (47.8)	1955 (26.3)	171 (17.5)	1381 (46.3)	428 (32.2)	4452 (32.2)
Prof. & Tech. & clerical	167 (34.4)	79 (16.6)	30 (14.6)	206 (42.4)	142 (29.6)	546 (28.9)
Sales	664 (39.2)	447 (20.3)	86 (16.0)	-	120 (23.5)	1317 (26.7)
Agric. & serv.	445 (45.9)	834 (22.6)	951 (20.3)	3165 (45.3)	913 (33.8)	5822 (33.3)
Manual	232 (39.4)	172 (22.0)	45 (16.8)	1104 (42.2)	293 (30.9)	2373 (33.4)
Others		41 (11.9)	-	-	-	41 (11.8)
Partner's Occup.						
Not working	--	228 (30.3)	11 (28.0)	38 (42.5)	53 (40.2)	329 (32.6)
Prof. & Tech. & clerical	166 (34.1)	124 (22.5)	51 (18.7)	228 (41.2)	181 (29.8)	749 (30.3)
Sales	137 (43.5)	152 (22.2)	38 (17.6)	-	42 (23.9)	370 (26.5)
Agric. & serv.	504 (44.1)	1726 (26.8)	552 (19.8)	2281 (45.9)	496 (32.4)	2289 (28.3)
Manual	477 (40.7)	230 (24.0)	146 (18.0)	1073 (43.6)	363 (30.3)	2289 (34.7)
Others	-	112 (26.7)	-	9 (53.1)	3 (31.4)	124 (27.7)
Parity						
0	641 (45.0)	862 (18.2)	456 (19.6)	1529 (46.1)	485 (31.7)	3394 (28.8)
1	264 (40.9)	396 (22.7)	170 (17.9)	989 (46.6)	284 (36.2)	849 (33.0)
2-3	498 (40.1)	696 (23.4)	302 (19.1)	1445 (43.2)	394 (28.3)	913 (30.0)
4-5	326 (40.9)	688 (28.4)	200 (19.4)	895 (41.8)	309 (30.2)	5071 (32.8)
≥6	238 (44.1)	885 (29.1)	157 (19.9)	997 (46.8)	426 (34.9)	2782 (34.7)
Age at 1^st^ birth						
<15	40 (27.9)	196 (25.4)	1 (3.3)	142 (47.0)	97 (31.4)	475 (30.9)
15-19	614 (43.6)	1532 (26.1)	230 (18.4)	2579 (45.1)	820 (31.2)	5775 (34.2)
20-24	487 (42.9)	747 (26.6)	450 (19.5)	1265 (42.2)	425 (32.9)	3373 (32.0)
25-29	142 (33.7)	154 (26.6)	122 (18.5)	277 (46.7)	64 (31.5)	760 (30.9)
≥30	44 (39.0)	37 (26.1)	26 (20.9)	64 (46.7)	8 (22.9)	4152 (29.9)
Bed net						
No	1186 (40.9)	-	470 (21.5)	2052 (40.5)	752 (34.9)	4459 (36.5)
Yes	782 (44.8)	-	815 (18.2)	3805 (47.2)	1146 (29.9)	6549 (36.1)
Contraceptive use						
Modern	310 (36.5)	737 (19.6)	280 (15.0)	1216 (34.3)	411 (24.5)	2953 (25.2)
Traditional	81 (39.5)	12 (17.1)	29 (15.4)	296 (43.1)	44 (23.1)	461 (34.4)
Intends to use later	556 (43.5)	1412 (22.8)	689 (20.7)	2439 (49.3)	926 (36.8)	6022 (33.0)
Not intend to use	1020 (44.1)	1367 (27.9)	287 (22.0)	1906 (49.2)	517 (32.2)	5097 (36.4)
Country						
Ghana						1,962 (42.3)
Ethiopia						3,527 (23.6)
Rwanda						1,284 (19.3)
Tanzania						5,857 (44.8)
Uganda						1,898 (31.7)

**(a):** 

Countries						
Predictive variables	Ghana 2014		Ethiopia 2016		Rwanda 2014-2015	
	CPRR	APRR	CPRR	APRR	CPRR	APRR
Age of Res.						
15-19	Ref.	Ref.	Ref.	Ref.	Ref.	Ref.
20-24	0.98 (0.87, 1.11)	1.07 (0.71, 1.60)	1.19 (1.03, 1.39)^∗^	0.98 (0.70, 1.37)	1.04 (0.88, 1.23)	1.04 (0.88, 1.25)
25-29	0.83 (0.72, 0.95)^∗∗^	0.93 (061, 1.42)	1.23 (1.06, 1.42)^∗∗^	0.81 (0.57, 1.16)	0.96 (0.81, 1.14)	1.02 (0.83, 1.25)
30-34	0.81 (0.70, 0.93)^∗∗^	0.85 (0.55, 1.31)	1.33 (1.15, 1.54)^∗∗∗^	0.74 (0.51, 1.08)	0.96 (0.80, 1.14)	1.05 (0.84, 1.32)
35-39	0.82 (0.71, 0.94)^∗∗^	0.83 (0.53, 1.29)	1.21 (1.03, 1.42)^∗^	0.62 (0.41, 0.92)^∗^	1.04 (0.86, 1.25)	1.16 (0.92, 1.47)
40-44	0.93 (0.81, 1.07)	0.89 (0.57, 1.41)	1.27 (1.07, 1.51)^∗∗^	0.61 (0.40, 0.92)^∗^	1.05 (0.86, 1.29)	1.11 (0.86, 1.44)
45-49	0.79 (0.66, 0.93)^∗∗^	0.75 (0.47, 1.20)	1.15 (0.94, 1.40)	0.52 (0.34, 0.79)^∗∗^	1.28 (1.05, 1.56)^∗^	1.28 (0.97, 1.69)
Residence						
Urban	Ref.	Ref.	Ref.	Ref.	Ref.	Ref.
Rural	1.03 (0.95, 1.12)	-	1.49 (1.33, 1.69)^∗∗∗^	1.15 (0.91, 1.44)	1.22 (1.07, 1.39)^∗∗^	1.14 (0.96, 1.35)
Res. Educ.						
No Educ.	Ref.	Ref.	Ref.	Ref.	Ref.	Ref.
Primary	0.98 (0.87, 1.10)	1.01 (0.87, 1.17)	0.78 (0.71, 0.86)^∗∗∗^	0.90 (0.78, 1.03)	0.85 (0.73, 0.99)^∗^	0.93 (0.79, 1.09)
Secondary	0.91 (0.82, 1.01)	0.95 (0.81, 1.09)	0.64 (0.54, 0.75)^∗∗∗^	1.12 (0.84, 1.48)	0.78 (0.65, 0.94)^∗∗^	0.94 (0.76, 1.15)
Higher	0.71 (0.55, 0.90)^∗∗^	0.79 (0.50, 1.25)	0.42 (0.32, 0.55)^∗∗∗^	0.43 (0.25, 0.76)^∗∗∗^	0.92 (0.68, 1.25)	1.25 (0.89, 1.73)
Wealth index						
Poorest	Ref.	Ref.	Ref.	Ref.	Ref.	Ref.
Poorer	1.16 (1.04, 1.30)^∗∗^	1.21 (1.04, 1.40)^∗^	0.74 (0.65, 0.84)^∗∗∗^	0.79 (0.68, 0.92)^∗∗^	0.81 (0.69, 0.94)^∗∗^	0.83 (0.71, 0.96)^∗^
Middle	1.04 (0.93, 1.16)	1.14 (0.96, 1.36)	0.69 (0.61, 0.79)^∗∗∗^	0.76 (0.67, 0.88)^∗∗∗^	0.75 (0.65, 0.89)^∗∗^	0.80 (0.68, 0.94)^∗∗^
Richer	0.85 (0.75, 0.97)^∗^	1.00 (0.81, 1.24)	0.61 (0.53, 0.69)^∗∗∗^	0.70 (0.59, 0.82)^∗∗∗^	0.65 (0.55, 0.77)^∗∗∗^	0.71 (0.51, 0.84)^∗∗∗^
Richest	0.87 (0.76, 0.99)^∗^	1.02 (0.80, 1.30)	0.51 (0.45, 0.58)^∗∗∗^	0.63 (0.50, 0.80)^∗∗∗^	0.67 (0.58, 0.78)^∗∗∗^	0.75 (0.62, 0.92)^∗∗^
Preg. at time of study						
No	Ref.	Ref.	Ref.	Ref.	Ref.	Ref.
Yes	1.06 (0.92, 1.22)	-	1.26 (1.08, 1.46)^∗∗^	1.03 (0.87, 1.22)	1.24 (1.03, 1.48)^∗^	1.07 (0.87, 1.31)
Health Ins.						
No	Ref.	Ref.	Ref.	Ref.		
Yes	0.97 (0.89, 1.05)	-	0.71 (0.57, 0.87)^∗∗^	0.91 (0.71, 1.17)	-	-
Marital status						
Never married	Ref.	Ref.	Ref.	Ref.	Ref.	Ref.
Married	0.91 (0.83, 1.00)	-	1.48 (1.32, 1.66)^∗∗∗^	-	0.88 (0.78, 0.99)^∗^	1.03 (0.88, 1.20)
Living with partner	0.96 (0.84, 1.09)	-	1.35 (0.91, 1.99)	0.97 (0.66, 1.42)	1.10 (0.95, 1.28)	1.19 (1.01, 1.42)^∗^
Widowed	0.94 (0.73, 1.22)	-	1.21 (0.90, 1.62)		1.44 (1.16, 1.79)^∗∗^	1.37 (1.07, 1.74)^∗^
Divorced	0.98 (0.78, 1.23)	-	1.07 (0.84, 1.36)		1.07 (0.78, 1.46)	1.03 (0.75, 1.43)
No longer living with partner	0.92 (0.75, 1.13)	-	1.55 (1.09, 2.22)^∗^	-	1.31 (1.02, 1.67)^∗^	1.27 (0.99, 1.64)
Partner's Educ.						
No Educ.	Ref.	Ref.	Ref.	Ref.	Ref.	
Primary	0.82 (0.68, 0.99)^∗^	0.85 (0.79, 1.03)	0.90 (0.81, 1.00)	1.03 (0.92, 1.17)	0.88 (0.74, 1.04)	-
Secondary	0.82 (0.73, 0.92)^∗∗^	0.88 (0.76, 1.02)	0.79 (0.66, 0.96)^∗^	1.07 (0.86, 1.35)	0.87 (0.67, 1.12)	-
Higher	0.86 (0.72, 1.03)	1.17 (0.87, 1.54)	0.64 (0.50, 0.81)^∗∗∗^	1.11 (0.81, 1.52)	0.81 (0.55, 1.19)	-
Do not know	0.88 (0.63, 1.24)	0.94 (0.66, 1.32)	1.28 (0.79, 2.07)	1.40 (0.89, 2.21)	1.22 (0.52, 2.83)	-
Woman's Occup.						
Not working	Ref.	Ref.	Ref.	Ref.	Ref.	
Prof. & Tech. & clerical	0.72 (0.59, 0.89)^∗∗^	1.02 (0.70, 1.48)	0.63 (0.48, 0.84)^∗∗^	1.65 (1.03, 2.63)^∗^	0.83 (0.59, 1.17)	-
Sales	0.82 (0.74, 0.91)^∗∗∗^	0.90 (0.76, 1.06)	0.77 (0.67, 0.89)^∗∗∗^	0.94 (0.79, 1.13)	0.92 (0.72, 1.16)	-
Agric.	0.96 (0.87, 1.07)	0.99 (0.83, 1.18)	0.86 (0.77, 0.96)^∗∗^	0.89 (0.79, 1.02)	1.16 (0.99, 1.35)	-
Services	0.82 (0.71, 0.95)^∗^	0.85 (0.69, 1.05)	0.84 (0.68, 1.02)	0.95 (0.73, 1.24)	0.96 (0.70, 1.31)	-
Others	-	-	0.45 (0.30, 0.67)^∗∗∗^	0.54 (0.29, 0.98)^∗^	-	
Partner's Occup.						
Not working	Ref.	Ref.	Ref.	Ref.	Ref.	.
Prof. & Tech. & clerical	-	-	0.74 (0.57, 0.98)^∗^	1.19 (0.89, 1.59)	0.65 (0.37, 1.15)	-
Sales	1.28 (1.02, 1.62)^∗^	1.45 (1.09, 1.93)^∗^	0.73 (0.57, 0.94)^∗^	0.95 (0.73, 1.24)	0.61 (0.34, 1.12)	-
Agric.	1.30 (1.09, 1.54)^∗∗^	1.30 (1.01, 1.67)^∗^	0.89 (0.75, 1.04)	0.98 (0.82, 1.15)	0.69 (0.41, 1.17)	-
Manual	1.20 (1.00, 1.44)^∗^	1.34 (1.06, 1.72)^∗^	0.79 (0.64, 0.99)^∗^	1.07 (0.85, 1.35)	0.63 (0.37, 1.08)	-
Others	-	-	0.88 (0.66, 1.17)	1.12 (0.83, 1.49)	-	-
Parity						
0	Ref.	Ref.	Ref.	Ref.	Ref.	
1	0.91 (0.79, 1.04)	-	1.25 (1.07, 1.46)^∗∗^	-	1.03 (0.98, 1.08)	-
2-3	0.89 (0.80, 0.99)^∗^	1.04 (0.86, 1.25)	1.29 (1.13, 1.47)^∗∗∗^	1.09 (0.90, 1.33)	1.02 (0.97, 1.07)	-
4-5	0.91 (0.81, 1.03)	1.11 (0.89, 1.39)	1.56 (1.37, 1.78)^∗∗∗^	1.48 (1.17, 1.86)^∗∗^	1.01 (0.99, 1.04)	-
≥6	0.98 (0.86, 1.11)	1.15 (0.89, 1.48)	1.60 (1.42, 1.81)^∗∗^	1.58 (1.21, 2.05)^∗∗^	0.99 (0.96, 1.03)	-
Age at 1^st^ birth						
<15	Ref.	Ref.	Ref.	Ref.	Ref.	
15-19	1.55 (1.14, 2.08)^∗∗^	1.58 (1.16, 2.16)^∗∗^	1.02 (0.83, 1.25)	-	5.54 (0.78, 39.24)	-
20-24	1.52 (1.13, 2.05)^∗∗^	1.64 (1.20, 2.25)^∗∗^	1.05 (0.84, 1.29)	-	5.87 (0.83, 41.43)	-
25-29	1.19 (0.85, 1.67)	1.49 (1.05, 2.14)^∗^	1.05 (0.79, 1.38)	-	5.59 (0.78, 39.63)	-
≥30	1.38 (0.93, 2.07)	1.69 (1.08, 2.64)^∗^	1.02 (0.65, 1.59)	-	6.30 (0.86, 45.75)	-
Bed net						
No	Ref.	Ref.			Ref.	Ref.
Yes	1.09 (1.01, 1.19)^∗^	1.05 (0.94, 1.17)	-	-	0.84 (0.76, 0.94)^∗∗^	0.92 (0.82, 1.04)
Contraceptive use						
Modern	Ref.	Ref.	Ref.	Ref.	Ref.	Ref.
Traditional	1.08 (0.84, 1.37)	1.27 (0.92, 1.75)	0.88 (0.43, 1.80)	1.09 (0.51, 2.29)	1.00 (0.0.69, 1.45)	1.05 (0.73, 1.51)
Intends later	1.19 (1.04, 1.36)^∗^	1.21 (1.03, 1.42)^∗^	1.17 (1.04, 1.32)^∗^	1.26 (1.09, 1.45)^∗∗^	1.38 (1.21, 1.58)^∗∗∗^	1.42 (1.22, 1.66)^∗∗∗^
Does not intend	1.21 (1.07, 1.37)^∗∗^	1.30 (1.12, 1.52)^∗∗^	1.43 (1.26, 1.60)^∗∗∗^	1.47 (1.28, 1.69)^∗∗∗^	1.47 (1.26, 1.72)^∗∗∗^	1.42 (1.19, 1.68)^∗∗∗^
Deviance goodness of fit test value		2085		6543		2388
*p* value of the chi-square		1.00		1.00		1.00

**(b):** 

Countries						
Predictive variables	Tanzania 2015-2016		Uganda 2016		All five countries	
	CPRR	APRR	CPRR	APRR	CPRR	APRR
Age of Res.						
15-19	Ref.	Ref.	Ref.	Ref.	Ref.	Ref.
20-24	0.97 (0.91, 1.04)	0.89 (0.80, 0.99)^∗^	1.02 (0.90, 1.16)	0.93 (0.77, 1.14)	1.04 (0.99, 1.09)	1.00 (0.87, 1.15)
25-29	0.91 (0.84, 0.98)^∗^	0.81 (0.72, 0.92)^∗∗^	0.83 (0.72, 0.96)^∗^	0.81 (0.65, 1.01)	0.94 (0.89, 0.99)^∗^	0.88 (0.76, 1.01)
30-34	0.86 (0.79, 0.94)^∗∗∗^	0.80 (0.75, 0.92)^∗∗^	0.94 (0.82, 1.09)	0.89 (0.72, 1.11)	0.96 (0.90, 1.01)	0.92 (0.79, 1.07)
35-39	0.97 (0.89, 0.94)	0.87 (0.75, 1.00)	0.94 (0.81, 1.10)	0.85 (0.68, 1.07)	1.00 (0.95, 1.07)	0.95 (0.81, 1.11)
40-44	0.95 (0.87, 1.04)	0.83 (0.72, 0.97)^∗∗^	1.02 (0.87, 1.19)	0.88 (0.68, 1.13)	1.06 (0.99, 1.12)	0.93 (0.78, 1.10)
45-49	0.91 (0.83, 1.00)	0.82 (0.69, 0.97)^∗^	0.98 (0.82, 1.18)	0.86 (0.66, 1.13)	1.00 (0.93, 1.07)	0.89 (0.73, 1.08)
Residence						
Urban	Ref.	Ref.	Ref.	Ref.	Ref.	
Rural	1.01 (0.96, 1.03)	-	1.21 (1.08, 1.36)^∗∗^	1.13 (0.95, 1.34)	0.97 (0.94, 1.02)	-
Res. Educ.						
No Educ.	Ref.	Ref.	Ref.	Ref.	Ref.	Ref.
Primary	0.86 (0.82, 0.92)^∗∗∗^	0.89 (0.83, 0.96)^∗∗^	0.86 (0.76, 0.98)^∗^	0.87 (0.74, 1.01)	0.96 (0.93, 1.00)	0.92 (0.82, 1.03)
Secondary	0.82 (0.75, 0.88)^∗∗∗^	0.84 (0.74, 0.95)^∗∗^	0.82 (0.71, 0.96)^∗^	0.97 (0.78, 1.19)	0.99 (0.93, 1.03)	0.89 (0.78, 1.01)
Higher	0.81 (0.60, 1.07)	0.92 (0.61, 1.39)	0.81 (0.66, 1.00)	0.95 (0.67, 1.34)	0.67 (0.59, 0.76)^∗∗∗^	0.87 (0.67, 1.13)
Wealth index						
Poorest	Ref.	Ref.	Ref.	Ref.	Ref.	Ref.
Poorer	0.95 (0.88, 1.02)	0.99 (0/91, 1.09)	0.81 (0.72, 0.91^)∗∗∗^	0.81 (0.69, 0.94)^∗∗^	0.87 (0.83, 0.92)^∗∗∗^	1.01 (0.88, 1.15)
Middle	0.95 (0.88, 1.01)	1.03 (0.94, 1.12)	0.76 (0.67, 0.85)^∗∗∗^	0.77 (0.65, 0.91)^∗∗^	0.84 (0.80, 0.99)^∗∗∗^	0.95 (0.83, 1.08)
Richer	0.85 (0.79, 0.91)^∗∗∗^	0.96 (0.87, 1.06)	0.78 (0.69, 0.88)^∗∗∗^	0.85 (0.71, 1.00)	0.77 (0.73, 0.81)^∗∗∗^	0.92 (0.81, 1.05)
Richest	0.90 (0.84, 0.97)^∗∗^	1.01 (0.90, 1.13)	0.62 (0.54, 0.71)^∗∗∗^	0.72 (0.58, 0.91)^∗∗^	0.73 (0.69, 0.77)^∗∗∗^	0.93 (0.81, 1.07)
Preg. at time of study						
No	Ref.	Ref.	Ref.	Ref.	Ref.	Ref.
Yes	1.31 (1.22, 1.40)^∗∗∗^	1.14 (1.05, 1.24)^∗∗^	1.23 (1.09, 1.39)^∗∗^	1.02 (0.88, 1.18)	1.27 (1.20, 1.34)^∗∗∗^	1.02 (0.92, 1.12)
Health Ins.						
No	Ref.	Ref.	Ref.	Ref.	Ref.	Ref.
Yes	0.86 (0.79, 0.95)^∗∗^	0.95 (0.84, 1.06)	0.89 (0.57, 1.39)	-	1.09 (1.04, 1.14)^∗∗∗^	0.91 (0.81, 1.03)
Marital status						
Never married	Ref.	Ref.	Ref.	Ref.	Ref.	Ref.
Married	1.02 (0.96, 1.07)	-	1.02 (0.91, 1.15)		1.08 (1.04, 1.13)^∗∗∗^	-
Living with partner	1.01 (0.94, 1.09)	-	1.01 (0.89, 1.14)	0.97 (0.86, 1.09)	1.19 (1.12, 1.26)^∗∗∗^	0.98 (0.90, 1.06)
Widowed	1.04 (0.90, 1.20)	-	1.36 (1.09, 1.69)^∗^		1.14 (1.03, 1.25)^∗^	1.19 (0.86, 1.67)
Divorced	1.09 (0.98, 1.21)	-	1.10 (0.71, 1.72)		1.07 (0.98, 1.18)	1.09 (0.81, 1.45)
Separated	0.98 (0.88, 1.11)	-	1.14 (0.97, 1.34)		1.24 (1.14, 1.34)^∗∗∗^	1.01 (0.78, 1.31)
Partner's Educ.						
No Educ.	Ref.	Ref.	Ref.		Ref.	Ref.
Primary	0.86 (0.79, 0.93)^∗∗∗^	0.95 (0.87, 1.03)	0.96 (0.78, 1.18)	-	0.99 (0.94, 1.05)	0.93 (0.81, 1.06)
Secondary	0.87 (0.78, 0.95)^∗∗^	0.95 (0.85, 1.08)	0.85 (0.67, 1.07)	-	1.04 (0.98, 1.11)	0.94 (0.81, 1.08)
Higher	0.82 (0.67, 1.00)	0.96 (0.76, 1.20)	0.83 (0.63, 1.08)	-	0.87 (0.78, 0.97)^∗∗^	1.04 (0.85, 1.28)
Do not know	0.84 (0.45, 1.53)	0.84 (0.42, 1.68)	0.93 (0.62, 1.38)	-	1.09 (0.89, 1.35)	1.02 (0.75, 1.38)
Woman's Occup.						
Not working	Ref.	Ref.	Ref.	Ref.	Ref.	Ref.
Prof. & Tech. & clerical	0.92 (0.79, 1.05)	0.89 (0.72, 1.10)	0.92 (0.75, 1.10)	0.96 (0.72, 1.27)	0.89 (0.81, 0.98)^∗^	0.93 (0.77, 1.11)
Sales	-	-	0.73 (0.59, 0.89)^∗∗^	0.69 (0.53, 0.89)^∗∗^	0.83 (0.77, 0.89)^∗∗∗^	0.79 (0.68, 0.90)^∗∗^
Agric. & serv.	0.98 (0.92, 1.03)	0.89 (0.82, 0.96)^∗∗^	1.05 (0.94, 1.17)	0.95 (0.81, 1.11)	1.03 (0.99, 1.08)	0.90 (0.81, 0.99)^∗^
Manual	0.91 (0.85, 0.98)^∗^	0.90 (0.81, 0.99)^∗^	0.96 (0.83, 1.10)	0.87 (0.71, 1.07)	1.03 (0.98, 1.09)	0.87 (0.79, 0.96)^∗∗^
Others	-	-				
Partner's Occup.						
Not working	Ref.	Ref.	Ref.	Ref.	Ref.	Ref.
Prof. & Tech. & clerical	0.95 (0.70, 1.29)	-	0.74 (0.56, 0.98)^∗^	0.92 (0.69, 1.24)	0.93 (0.81, 1.07)	1.03 (0.70, 1.52)
Sales	-	-	0.59 (0.41, 0.86)^∗∗^	0.78 (0.53, 1.13)	0.81 (0.69, 0.96)^∗^	1.22 (0.79, 1.86)
Agric.	1.06 (0.80, 1.41)	-	0.81 (0.63, 1.04)	0.87 (0.66, 1.13)	0.87 (0.76, 0.98)^∗^	1.08 (0.70, 1.65)
Manual	1.01 (0.75, 1.34)	-	0.75 (0.58, 0.97)^∗^	0.91 (0.69, 1.19)	1.06 (0.93, 1.21)	1.11 (0.73, 1.68)
Others	1.23 (0.67, 2.26)	-	0.77 (0.28, 2.13)	0.91 (0.31, 2.69)	0.85 (0.66, 1.09)	2.00 (0.85, 4.66)
Parity						
0	Ref.	Ref.	Ref.	Ref.	Ref.	Ref.
1	1.01 (0.94, 1.09)	1.04 (0.93, 1.18)	1.14 (0.99, 1.31)	-	1.14 (1.05, 1.24)^∗∗∗^	0.96 (0.72, 1.28)
2-3	0.94 (0.88, 1.00)	0.99 (0.87, 1.13)	0.89 (0.79, 1.02)	-	1.04 (0.96, 1.13)	0.92 (0.68, 1.23)
4-5	0.91 (0.84, 0.98)^∗^	1.02 (0.87, 1.13)	0.95 (0.83, 1.09)	-	1.14 (1.09, 1.19)^∗∗∗^	0.97 (0.82, 117)
≥6	1.01 (0.94, 1.09)	1.09 (0.95, 1.28)	1.07 (0.95, 1.21)	-	1.20 (1.14, 1.27)^∗∗∗^	-
Age at 1^st^ birth						
<15	Ref.	Ref.	Ref.	Ref.	Ref.	Ref.
15-19	0.96 (0.82, 1.11)	-	0.99 (0.82, 1.21)	-	1.11 (0.99, 1.23)	-
20-24	0.89 (0.77, 1.05)	-	1.05 (0.85, 1.29)	-	1.04 (0.93, 1.15)	-
25-29	0.99 (0.83, 1.19)	-	0.99 (0.74, 1.34)	-	1.00 (0.88, 1.14)	-
≥30	0.99 (0.76, 1.29)	-	0.73 (0.34, 157)	-	0.97 (0.87, 1.08)	-
Bed net						
No	Ref.	Ref.	Ref.	Ref.	Ref.	Ref.
Yes	1.15 (1.09, 1.21)^∗∗∗^	1.21 (1.13, 1.29)^∗∗∗^	0.86 (0.79, 0.93)^∗∗∗^	0.91 (0.81, 1.02)	0.99 (0.96, 1.03)	-
Contraceptive use						
Uses modern contraceptive	Ref.	Ref.	Ref.	Ref.	Ref.	Ref.
Uses traditional method	1.25 (1.11, 1.42)^∗∗∗^	1.37 (1.19, 1.58)^∗∗∗^	0.94 (0.69, 1.29)	1.02 (0.73, 1.43)	1.36 (1.23, 1.51)^∗∗∗^	1.22 (1.03, 1.16)^∗^
Nonuser intends to use later	1.44 (1.34, 1.53)^∗∗∗^	1.48 (1.36, 1.61)^∗∗∗^	1.49 (1.34, 1.68)^∗∗∗^	1.44 (1.25, 1.67)^∗∗∗^	1.31 (1.25, 1.37)^∗∗∗^	1.51 (1.36, 1.67)^∗∗∗^
Does not intend to use	1.43 (1.34, 1.53)^∗∗∗^	1.51 (1.38, 1.64)^∗∗∗^	1.31 (1.15, 1.49)^∗∗∗^	1.32 (1.12, 1.56)^∗∗^	1.44 (1.37, 1.51)^∗∗∗^	1.41 (1.26, 1.57)^∗∗∗^
Countries						
Ghana	-	-	-	-	Ref.	Ref.
Ethiopia	-	-	-	-	0.56 (0.52, 0.59)^∗∗∗^	0.62 (0.56, 0.69)^∗∗∗^
Rwanda	-	-	-	-	0.45 (0.43, 0.48)^∗∗∗^	-
Tanzania	-	-	-	-	1.06 (1.01, 1.11)^∗^	1.10 (0.99, 1.20)
Uganda	-	-	-	-	0.75 (0.71, 0.79)^∗∗∗^	0.77 (0.69, 0.85)^∗∗∗^
Deviance goodness of fit test value		5201		2397		11136
*p* value of the chi-square		1.00		1.00		1.00

Res.: respondent; Educ.: education; Occup.: occupation; Prof.: professional; serv.: services; Agric.: agricultural; Preg.: pregnant; Ins.: insurance; CPRR: crude prevalence rate ratio; APRR: adjusted prevalence rate ratio; Ref.: reference; ^∗^*p* < 0.05, ^∗∗^*p* < 0.01, and ^∗∗∗^*p* < 0.001.

## Data Availability

An application requesting for the use of the Demographic and Health Surveys data was sent to the DHS website. Data was then used after approval was obtained. The datasets generated and/or analyzed during the current study are available in the Demographic and Health Survey Repository, http://dhsprogram.com/data/available-datasets.cfm.
